This article has been retracted.

# Impact of artificial light intensity on nocturnal insect diversity in urban and rural areas of the Asir province, Saudi Arabia

**DOI:** 10.1371/journal.pone.0242315

**Published:** 2020-12-01

**Authors:** Abdulrahim Refdan Hakami, Khalid Ali Khan, Hamed A. Ghramh, Zubair Ahmad, Adil Ali Ahmad AL-zayd

**Affiliations:** 1 Department of Clinical Laboratory Sciences, College of Applied Medical Sciences, King Khalid University, Abha, Saudi Arabia; 2 Research Center for Advanced Materials Science (RCAMS), King Khalid University, Abha, Saudi Arabia; 3 Unit of Bee Research and Honey Production, Faculty of Science, King Khalid University, Abha, Saudi Arabia; 4 Biology Department, Faculty of Science, King Khalid University, Abha, Saudi Arabia; 5 Biology Department, Faculty of Sciences and Arts, King Khalid University, Dhahran Al-Janoub, Saudi Arabia; Harran University, TURKEY

## Abstract

Continuous urban developments have resulted in increased demand for street furniture, one of which is street light columns. Artificial light at night (ALAN) pose significant impacts on insect diversity in urban and rural areas. The ALAN is a significant driver of decline in insect diversity. This study evaluated the impact of light intensity and sky quality at night on insect diversity in rural and urban areas of the Asir province, Saudi Arabia. Insect traps were installed in both areas during night. Light intensity of nearby road lamps was measured using light meter, while sky quality was measured using sky quality meter. Rural areas exhibited low light intensity (10.33 flux/f.candle) and good sky quality (18.80 magnitude/arcsec^2^). Urban areas exhibited intense light (89.33 flux/f.candle) and poor sky quality (15.49 magnitude/arcsec^2^). Higher insect diversity was recorded for rural areas where insects belonging to seven orders (i.e., Diptera, Lepidoptera, Hemiptera, Hymenoptera, Coleoptera, Neuroptera, and Dermaptera) were collected. However, insects of four orders (i.e., Diptera, Lepidoptera, Hemiptera, and Neuroptera) were found in urban areas indicating low diversity. Lepidopteran insects were frequently recorded from rural areas indicating they are attracted to artificial light. It is concluded that excessive ALAN and poor sky quality at night disrupt insect biodiversity. Therefore, ALAN and sky quality must be considered responsible for decline in insect biodiversity along with other known factors.

## Introduction

Global insect diversity is declining and >40% of the world's insect species could go extinct over the next several decades if declining trends are not halted/reversed [1]. The most common drivers of these declines are intensive agriculture, excessive pesticide use, urbanization, climate change and habitat destruction [1, 2]. Dramatic loss of insect diversity in many parts of the world has attracted the attention of scientists to consider detrimental impacts on human health and livelihoods. Drastic decline of flying insects “Ecological Armageddon” was reported by Hallmann et al. [3]. Malaise traps were used by Hallmann et al. [3] to collect data from an agricultural landscape and >75% decline in insect biomass was recorded over 27 years. This study on decline in insect biodiversity gained significant attention in the scientific community. The substantial loss of insect populations can not only be explained by changes in habitat, climate or land use [3], but there are some other large-scale factors which could also be involved.

According to Grubisic et al. [2], artificial light could be an overlooked driver of insect declines. Urbanization has resulted with a new phenomenon associated with cities and towns called ‘light pollution” [4], which has significant impact on animals and insects throughout the world [5]. Increasing artificial light at night (ALAN) is the primary cause of this phenomenon. It is mainly connected to general population growth, industrial development and rising economic prosperity. Installation of lamps with higher luminous efficiency has also played a negative role in insect diversity declines.

The ALAN is known to have strong impacts on population dynamics of insects. Globally it has been increasing at an annual rate of 2%–6% over the last decades [6, 7], imposing an unprecedented alteration of natural light regimes and threatening biodiversity [8]. Despite its ubiquity, the importance of artificial light as an agent of global change is often overlooked when analyzing insect population declines. Insects perform many functions and provide essential support in agroecosystems. They provide ecosystem regulation services such as decomposition of organic material, nutrient and energy flow regulation, seed and pathogen dispersal, pollination, control of pests and conservation of biodiversity [9]. Therefore, decreasing number of insects may substantially affect maintenance of these functions and services, with consequences for food production and biodiversity health. Light is an important visual and non-visual cue for insects [10]. More than 60% of all invertebrates are nocturnal [8] and utilize nocturnal light for orientation, navigation, avoidance of predators, location of food and reproduction [11]. Many nocturnal and crepuscular insects use celestial light sources such as stars and the moon as visual cues for dispersal across landscapes [12].

The effect of sky quality and light intensity on nocturnal insects have never been studied in Saudi Arabia. The aim of this study was to examine the impact of ALAN on insect diversity in rural and urban areas. We emphasized the impact of artificial light on insects and compared the effect of sky quality at night and light intensity on nocturnal insects both in urban and rural areas of Saudi Arabia. We investigated the impact of ALAN on insect population declines in light-polluted areas and rural agricultural areas.

## Materials and methods

The experiment was set up according to Manfrin et al. [13] with some modifications. Data relating to diversity of nocturnal flying insect in rural and urban sites were collected to evaluate the impact of light intensity and sky quality on insect diversity in rural and urban areas.

### Study area

This field experiment was conducted in Asir province, Saudi Arabia. No specific permits were required to execute this study and the work did not involve any endangered species. Two different locations, i.e., Mohayil and Abha were selected for this study. We delimited locations according agricultural (Mohayil) and urban area (Abha). Mohayil is characterized by an agricultural landscape, whereas Abha is an urban area. An agricultural farm in Mohayil (18° 12ʹ 24.76ʺ N; 42° 32ʹ 17.51ʺ E) with no prior exposure to artificial light and another location in Abha city (18° 31ʹ 45.31ʺ N; 42° 2ʹ 42.95ʺ E) with light exposure were selected.

### Environmental conditions

Data were collected during February and March, 2020. Light intensity was measured in lux through a light meter, Digitech, QM1587 (Reduction Revolution Pty Ltd, Parramatta, Australia) (Fig 1A). The light meter reads ambient light or direct light from an artificial source and calculates the correct shutter speed and aperture values required to capture an accurate exposure. The sky quality was measured in visual magnitudes per square arc second (magnitude/arcsec^2^) using sky quality meter (Unihedron, Ontario, Canada) (Fig 1B). Readings of the sky quality meter are inversely proportional to light; hence, higher digits indicate less light intensity. We compared sky quality measurements at different sites quantitatively.

**Fig 1:** Devices used in the experiment. (A) light meter to measure the light intensity from nearby street lights, and (B) sky quality meter to determine the darkness of sky at night.

### Insect collection and identification

Insects were collected from both sites using DynaTrap insect trap (Dynamic Solutions/MII Equipment Inc. Milwaukee, USA). It collects nocturnal flying insects including mosquitoes. Its ultraviolet light and whisper-quiet fan attracts and captures insects without zapping or buzzing. The trap does not use pesticides or chemicals or need an attractant or propane (Fig 2A). Traps were installed from evening to morning (19:00 to 7:00 local time) on every Thursday to Saturday. Sampling was carried out weekly during 1^st^ February to 31^st^ March 2020. The collected specimens were stored in papilon paper in the multipurpose plastic boxes and brought to laboratory for pinning and identification. Order level identification was primarily based on the description by Johnson and Triplehorn [14]. The collected specimens were kept in the Zoological Museum of the College for future reference (Fig 2B and 2C).

**Fig 2:** Experimental steps. (A) DynaTrap insect trap for insect collection, (B) insect trap installed at a rural site and (C) counting and identification of captured insects.

### Statistical analysis

Data were analyzed using the ‘pacman’ package Rinker et al. [15] in R (version 3.6.3; R Core Team, 2019). The analysis included boxplot structure, scatter plot and summary. Only night samples were analyzed for the comparisons of artificial light intensity and sky quality.

## Results

### Environmental conditions and measurements

Temperature, relative humidity, sky quality and light intensity were 26 to 27°C, 62% to 63%, 18.09 to 19.20 magnitudes/arcsec^2^ and 10 to 11 flux/f.candle, respectively in rural area. Similarly, a temperature between 18 and 19°C, 70% to 74% relative humidity, 15.18 to 16.10 magnitudes/arcsec^2^, and 88 to 90 flux/f.candle were recorded for urban area. The altitude of rural area was 530 m above sea level, while urban area is located at an elevation of 2215 m. Table 1 summarizes environmental data of both experimental sites. A significant difference (*p* ≤ 0.05) was observed in all environmental variables, i.e., light intensity, sky quality, altitude, relative humidity and temperatures between rural and urban area.

**Table 1:** Environmental data of rural and urban sites included in the study.

Location	Light Intensity (flux/f.candle)	Sky quality (msgs/arcsec^2^)	Altitude (m)	Relative Humidity (%)	Temperature (°C)
Mohayil (rural)	10.33 ± 0.58^**B**^	18.80 ± 0.61^**B**^	530 ± 0.0^**B**^	62.33 ± 0.58^**B**^	26.67 ± 0.58^**B**^
Abha (urban)	89.33 ± 1.15^**A**^	15.49 ± 0.53^**A**^	2215 ± 0.0^**A**^	72.33 ± 2.08^**A**^	18.67 ± 0.58^**A**^

Means followed by same letters within a column are statistically non-significant.

Light intensity at night was high (89.33 flux/f.candle) with low sky quality (15.49 msgs/arcsec^2^) in urban area. On the other side, rural area recorded limited manmade intervention (10.33 flux/f.candle) and better sky quality (18.80 msgs/arcsec^2^) (Fig 3).

**Fig 3:** Scatter plot showing the relationship between light intensity and sky quality at rural and urban areas.

### Diversity of nocturnal flying insects

The insect traps installed at both areas collected insects belonging to seven different orders. Insects from rural site belonged to Diptera, Lepidoptera, Hemiptera, Hymenoptera, Coleoptera, Neuroptera, and Dermaptera orders. The insects collected from urban area belonged to four orders namely Diptera, Lepidoptera, Hemiptera and Neuroptera. The number of insects collected from Diptera, Lepidoptera, Hemiptera, Hymenoptera, Coleoptera, Neuroptera, and Dermaptera orders ranged between 0–43, 37–156, 0–55, 0–5, 11–66, 0–2 and 0–7, respectively in rural area. Similarly, 1–9, 2–9, 0–1 and 0–2 insects were collected for Diptera, Lepidoptera, Hemiptera and Neuroptera, respectively from urban areas.

The average number of insects collected from rural area in orders Diptera, Lepidoptera, Hemiptera, Hymenoptera, Coleoptera, Neuroptera and Dermaptera were 18.67, 89.67, 22.00, 1.67, 30.67, 1.00 and 3.00, respectively. In urban area average number of insects belonging to Diptera, Lepidoptera, Hemiptera and Neuroptera were 5.33, 5.00, 0.33 and 0.67, respectively (Fig 4). Lower population of Lepidopterans in urban area suggests that these insects were attracted to the uncountable number of the city white light LEDs. The peak of Lepidopteran insects’ attraction is attained when blue or white light emits shorter wavelengths around 400 nm [16]. It has been observed in Abha that a huge number of insects were attracted to newly-lit areas that have not been lit before. This attracts bats to feed on them. No attraction was observed to the high pressure sodium lamps within the city that are still installed in many roads, although white LEDs are now increasing in an alarming rate.

**Fig 4:** Box plot showing the population of insect orders in response to light intensity and sky quality. (A) box plot for insect diversity in rural area and (B) box plot for insect diversity in urban area.

## Discussion

Nocturnal insects are highly sensitive to light and their behavioral responses like dispersal, foraging, defense against predation, location of food, hosts, oviposition sites, resting sites and mate searching are governed by vision [17–25]. These behavioral responses of insects are very much related with light intensity (adaptation), circadian periodicity and photoperiodism [20, 24]. Nocturnal behavior of insects, their growth and physiology can be disrupted by the use of artificial light at night (ALAN) [23, 24]. However, the reason for this phototactic behavior, especially for ALAN in nocturnal insects remains unclear and may be driven by multiple factors [18, 20, 26]. The effects of environmental (e.g. light intensity, exposure time of light, polarization, weather and season) and physiological (e.g. sex, mating status, age and adaptation to the dark) factors as well as other anthropogenic activities (e.g. intensive agricultural practices), which leads are prominent examples that may affect insect’s population in rural and urban areas [27, 28]. As a consequence, long-term exposure of nocturnal insect communities to ALAN can lead to changes compared to communities that are less exposed to light [29, 30]. Most of the studies on the effect of light intensities have focused on birds, larger vertebrate animals and only a few studies have devoted on insect population affection light intensities. This is first study in the kingdom of Saudi Arabia investigating the impact of ALAN on nocturnal flying insects in urban and rural areas. The current study confirmed our hypothesis that sky quality and artificial light intensity influences composition and abundance of the insects. Phototactic behavior of insects is also affected by sky quality, light quality and external shape of light source [17, 18, 21, 31]. Species diversity and abundance of insects caught by light traps can change according to the light source, for example, LED bulb, compact fluorescent bulb or incandescent bulb [31]. In rural area sky was clear and light intensity from artificial sources was lower than urban areas. This phenomenon proved good for insect diversity and populations [17, 18, 21]. Indeed, natural areas with low-level of artificial light are valuable to maintain healthy ecosystem and balanced insect diversity. In rural area seven insect orders were observed compared to four insect orders in the urban area. Artificial illumination attracted large number of nocturnal flying insects. Light sources function as an ecological trap [32] for many insects. This occurs during swarming events, when very large numbers of population are attracted to artificial light sources [33]. If not killed immediately, insects are often unable to disperse and migrate elsewhere [32, 34]. Several studies have shown how artificial illumination disrupts dispersal patterns in arthropods, confounding natural sources of orientation (e.g., moonlight) and attracting positively phototactic insects [35, 36]. In this study, majority of insects collected in the light traps were of nocturnal nature suggesting that these might be sensitive; thus, more vulnerable to light intensity [37]. In urban areas, increased light intensity at night distracts significant number of insects. This could be a possible reason for the low diversity and the reduced number of insets. These results are in accordance with Horváth et al. [35], Meyer and Sullivan [36]. Moreover, the presence of artificial light may affect the distance that organisms and nocturnal creatures move away [34, 38]. The ALAN has substantial effects on insect fauna, including moths. Macgregor et al. [39] reported that moth abundance was reduced to half and flight activity was 70% greater at lit sites as compared to dark areas. They further reported a considerable reduction in pollen transport by moths at areas with artificial light. Their findings supported the disruptive impact of ALAN on moth activity, which is a one proposed mechanism driving moth declines, and suggest that street lighting may potentially affect pollination of nocturnal invertebrates. In our study, the lepidopteron insects were significantly higher in an agricultural farmland (that has not experienced lighting projects before) than urban area. These findings are in agreement with Macgregor et al. [39] who reported that street lights have disruptive impact on moth behavioral activities. Considering the overall scenario, our results demonstrate that the intensity of light in urban environment might be a potential threat to the nocturnal insects’ diversity.

## Conclusions

Natural darkness at night is beneficial for insect species and entire wildlife. This may be understood by the high diversity of insects in rural areas. On the other hand, well-lit areas at night would negatively affect insect population, and this has been proved in this study. The right type of light and the intensity required for urban life are suggested to be considered carefully. Warm light that emits the wavelengths of yellow light may reduce some of the negative impacts and can reduce the number of insects attracted to irresistible artificial light.
